This article has been retracted.

# Application of Low-Intensity Laser in the Treatment of Skeletal Muscle Injury in Runners

**DOI:** 10.1155/2022/1211602

**Published:** 2022-06-17

**Authors:** Youdong Chen, Qiang Li

**Affiliations:** ^1^School of Clinical Medicine, Hunan University of Chinese Medicine, Changsha 410000, Hunan, China; ^2^Hunan University of Chinese Medicine, Hunan Province Second People Hospital, Changsha 410000, Hunan, China

## Abstract

With the continuous improvement of people's economic level, running, as the most common sports, is not limited by sports venues and sports levels and deeply loved by people. However, during running, soft tissue resonates with the impact force, increasing the load on joints and tendons and potentially leading to sports injuries. The purpose of this article is to study the application of low-intensity laser in the treatment of muscle strain. This article analyzes running, muscle adjustment, and lower limb stiffness. On the basis of theory, 20 healthy male college students were selected as research objects in the experimental part. The subjects were allowed to run at three speeds: slow, medium, and fast. The kinematics, dynamics, and surface EMG signals of the subjects during running were collected to analyze the effect of low-intensity laser therapy on exercise muscle strain. The experimental results showed that a low-intensity laser can effectively alleviate muscle inflammation, reduce the number of cell damage, bring the mean and integral optical density of protein to the normal level significantly, and reduce the strain degree of exercise muscle. In this article, a statistical method was used to obtain the gait cycle time (P & LT; 0.01) and support cycle time (slow *P* < 0.01).

## 1. Introduction

With the continuous development of China's society and economy and the continuous improvement of people's requirements for quality of life, a healthy and high quality of life has become a lifestyle that people increasingly pursue. At the same time, the three high issues caused by obesity and poor living habits are seriously affecting people's health. Therefore, fitness has changed from the earlier emerging things to the normal state of people's daily life. Physical fitness can not only beautify the appearance of the body but also improve the regulation of the nervous system and promote the growth of bones and muscles. Among many fitness methods, running is widely accepted by the general public because of its simple technical requirements and not being restricted by too many venues, clothing, and equipment and has become an important fitness method. Running can enhance the body's metabolism and basal metabolic rate and has a good effect on weight loss, fat loss, exercise, and enhancement of body immunity, antiviral ability, and resistance. Running for a long time is a very effective aerobic exercise, which can have a good effect on the cardiovascular endothelial system and can effectively reduce the incidence of coronary atherosclerotic heart disease, acute stroke, cerebral infarction, and other serious cardiovascular and cerebrovascular diseases. Regular running can also reduce blood lipids and can significantly reduce the concentration of triglycerides, cholesterol, uric acid, and blood sugar, so it has a good effect on the prevention and healthcare of the above diseases. Long-term running will play a certain role in promoting and regulating gastrointestinal digestion and absorption and effectively improve sleep and the sleep quality of the human body.

In normal human movement, factors such as running speed, distance, and frequency are usually determined or selected by the athlete at will. Everyone has their own suitable frequency, and the impact of this suitable frequency on human soft tissue is different. In this article, the effects of running frequency on stiffness and muscle tuning of the lower limbs are analyzed using microscope-based medical imaging diagnostic technology, simultaneous acquisition of dynamics and kinematics, and surface electromyography data. It provides a theoretical basis for people to choose a reasonable running frequency when running.

The purpose of Park et al. is to enable anyone to semiautomatically segment anatomical structures in MRI, CT, and other medical images on a personal computer. When performing semiautomatic segmentation in Adobe Photoshop, appropriate algorithms can be used, the degree of automation can be adjusted, a convenient user interface can be used, and software errors rarely occur [1]. Bailey's team aimed to compare the relationship between stride length (SL), stride frequency (SF), and speed when running on a treadmill and on the ground. Strategies for changing SL across speeds are different on treadmills and on the ground [2]. Faber and his team, due to their junior grades having little predictive value for future success, sought other solutions to assess the potential of young players. The purpose of this systematic review is to outline the tools that measure the personal determinants of young athletes in racket sports and to evaluate the effectiveness of these tools on talent development. The lack of longitudinal research makes it impossible to validate the instrument's ability to predict future performance [3].

In this article, 20 ordinary healthy male college students were selected as the research object, and the subjects were subjected to slow, medium, and fast. This kind of speed is used to run, and the kinematics, dynamics, and surface EMG signals of the subjects during running are collected simultaneously. In each speed mode, the subjects were divided into a low-cadence group and a high-cadence group; the stiffness of the lower limbs in the buffer phase and the active kick-extension phase were calculated based on the vertical reaction force peaks in the support phase and the vertical displacement of the center of gravity. Muscle vibration frequencies were analyzed prior to landing to analyze muscle tuning to analyze the effect of low-intensity laser therapy on exercise muscle strain [4].

## 2. Proposed Method

### 2.1. Lower Limb Stiffness

Stiffness is a physical term that refers to the ability of an object to resist deformation when it is loaded. The greater the stiffness of an object, the smaller its deformation [5]. For the human body, its stiffness value determines the strength of the supporting tissue and the body's ability to resist external forces. Generally speaking, the individual stiffness value is determined by muscles, tendons, ligaments, and bones. You can use a spring to simply show the relationship between the external force acting on the system and causing displacement. It will be found that under external force, the change in the displacement of the spring has a linear relationship with the applied external force, which is called the spring-mass model [6, 7]. For the human body, its overall skeletal muscle system also has elastic characteristics, which will change in length with external forces. In engineering applications, the stiffness of the structure is very important, so the elastic modulus is an important indicator when selecting materials. A high modulus of elasticity is necessary when there is an unpredictably large deflection. When the structure needs to have good flexibility, the elastic modulus is not required to be too high [8].

The elastic characteristics of the human skeletal muscle system are similar to springs. The self-regulation mechanism of human muscle stiffness helps the body better adapt to the external environment and can effectively maintain the stability of body posture [9, 10]. However, unlike the simple spring-mass model in the sense of general physics, a spring-mass model that can effectively restore the state of human movement should be able to integrate various soft tissue components, including human bones, muscles, tendons, and cartilage, and can contain biological tissue viscosity, muscle reflex time, central nervous system control, and many other factors. Obviously, the simple spring-mass model cannot take all the above factors into account. Therefore, this simple spring-mass model commonly used in the field of biomechanics to evaluate the stiffness of lower limbs is called quasistiffness.

In the field of biomechanics, the stiffness of lower limbs that people study can usually be divided into three types: vertical stiffness, leg stiffness, and joint stiffness. They have different ranges of action. In actual scientific research, vertical stiffness is mostly used to study vertical movements such as straight knee bouncing and jumping. The calculation method is to divide the peak vertical reaction force from the ground by the body divided by the vertical displacement distance of the center of gravity of the body; use vibration period and body mass to calculate by formula *K*=*m*(2*π*/*p*)^2^ (*p* is the period of vertical vibration) or calculate the natural frequency of vibration according to the landing time and the vacant time between continuous movements, and then use the formula *K*=*mω*^2^ to calculate the lower limb stiffness (*m* is the body mass and *ω* is the natural frequency of vibration). Leg stiffness is mainly used to describe walking or running. The calculation of leg stiffness is often performed using McMahon's formula *K*=*F*/Δ*L*. F is the maximum vertical reaction force from the ground received by the lower limbs and Δ*L* is the maximum vertical displacement distance of the center of gravity of the body during the movement; joint stiffness is biased to describe the rotation characteristics of the joints during the lower limb movements. The change in joint torque is usually divided by Change (*K*=Δ*M*/Δ*θ*, whereΔ*M* is the change in joint torque and Δ*θ* is the change in joint angle).

When the human body is performing a deep jump, the sensory system can sense the stretch load and falling height of the limbs, thereby acting on the neuromuscular system of the human body and judging the ground conditions during landing by the visual system, thereby activating the functional muscle groups in advance and making the human body better adapted to sports surfaces. That is, in the movement, when the human body makes reasonable judgments on the ground conditions through feedback from the visual system and commands from the central nervous system, the muscles are adjusted to a suitable stiffness before landing, and when the muscles are eccentrically contracted, they are obtained by stretch reflection. After better activity, the muscle will be preactivated, and this phenomenon will be reflected in myoelectric activity. This regulating ability has been discovered by scientists and is considered to be an important mechanism for regulating the stiffness of the lower limbs to prevent sports injuries.

In addition, the regulation of human lower limb stiffness is also related to age. When performing the action of descending stairs, the lower limb joint angle of the elderly is smaller and the muscle stiffness is greater; when performing the vertical jump in place, the elderly have worse muscle strength and lower limb stiffness adjustment ability than those of the young adults. It is believed that the ability of self-regulation during muscle contraction will decrease with aging [11].

There is also a correlation between the stiffness of the lower limbs and the hardness of the moving surface. The stiffness of the lower limbs of the human body when running in soft shoes is greater than the stiffness of the lower limbs when wearing hard shoes. During exercise, the lower limbs can perform a series of self-regulation according to the ground conditions so that the human body can better adapt to the ground hardness and achieve an optimal lower limb-ground overall stiffness value, which also shows that the human body will use the sensory motor function system to exercise. The hardness of the surface is appropriately adjusted so that the body can maintain the accuracy and balance of movements on the ground with different hardness. The stiffness of the lower extremity when jumping on the softest sports surface is twice that of the hardest sports surface, and the stiffness of the ankle joint and the extent of knee straightening also increase. It can be seen that the adjustment of lower limb stiffness in human movement is closely related to the adjustment of limb position and joint angular stiffness. It is often necessary to adjust the joint angular stiffness and limb position to adapt to the condition of the sports surface so that the body maintains the same posture on different sports surfaces [12].

### 2.2. Muscle Tuning

During exercise, the soft tissue structure of the human body (muscles, tendons, fascia, surrounding tissues, and skin) has a certain natural frequency and has the characteristic of changing its own frequency with changes in exercise state (systolic, diastolic, and forced conditions) [13]. In the study of impact force, we can consider the soft tissue structure, including muscles, tendons, fascia, and skin, as a vibration system, and the impact force as a set of input signals from the outside has the characteristics of causing soft tissue to vibrate. When the frequency of the impact force from the outside is close to the natural frequency of the soft tissue, the muscle will have a resonance phenomenon, which will increase the amplitude, but this phenomenon will disappear after the soft tissue vibrates twice. This is a muscle tuning activity performed by the human body in order to avoid soft tissue resonance leading to sports injuries; it can reduce the frequency of muscle vibrations and avoid sports injuries [14].

It can be seen that before the human body performs a series of running and jumping movements, the neuromuscular system will preactivate according to the landing conditions (such as ground hardness and speed of movement) and will reduce the frequency of soft tissue vibration through its own muscle tuning mechanism to avoid sports injuries. This process is called muscle tuning [15, 16]. The purpose of muscle tuning is to prevent the occurrence of resonance phenomenon caused by the external input frequency being close to its own natural frequency during exercise so as to prevent sports injuries and helps the repair of muscles and tendons; stretching exercises can stretch muscles and tendons, help prevent muscle tension, and relieve muscle soreness that often occurs after intense exercise [17]. During the muscle tuning process, the human body adjusts joint stiffness and joint position, thereby activating the soft tissues involved in movement and avoiding resonance. In general, during the entire exercise of the human body, the preactivation phenomenon will occur before the muscles touch the ground. At the same time, the joint stiffness and joint position of the human body will change accordingly during exercise. This series of adjustments is the performance of muscle tuning. The purpose is to reduce resonance, adapt to the state of exercise, and avoid sports injuries [18].

Muscles adjust vibration in the workplace; that is, when muscles encounter the potential danger of resonance, they adjust themselves to avoid resonance. During the movement of the human body, the active state of the lower limb muscles will change with the change of the impact force. When the frequency of the impact force from the outside in the exercise is close to the natural frequency of the quadriceps, the preactivation of the muscle will be significantly enhanced. In addition, when the human body moves without predicting the condition of the sports surface, the adjustment of the muscles when they touch the ground will change greatly. In this state, when the input frequency is close to the natural frequency, the resonance effect of the muscle will be more obvious. During the pretouchdown phase of human movement, muscle activity is mainly preparing for the next movement. The degree of muscle activation at this time is the impact force (including vibration frequency and amplitude) received by the previous muscle.

Moreover, muscle tuning is a holistic concept. It is a series of adjustments made by the muscles to avoid resonance, including changes in the geometric position of the lower limbs, changes in the stiffness of the lower limbs; adjustment of the vibration frequency of the soft tissues, changes in the load of the joints of the lower limbs, stability during the support phase, and action advancement during the off-ground phase.

### 2.3. Running

Running is a kind of periodic motion in which one-leg support alternates with vacancy, step-and-swing coordination, and coordinated and coherent movements. It is one of the main ways for the human body to complete displacement, and it is also a natural movement of human body movement. The human body experiences two single-leg supports and two emptyings in a running cycle. The support period is from the time when the foot hits the ground to the time when the foot is off the ground, including the front support stage and the rear kick stage, and the vacant period is from the time when one foot is off the ground to the time when the other foot is touched, including the back swing stage and the front swing stage. Running uphill (downhill) can stimulate the calf muscles, allowing rapid muscle strength growth. Fast running is an anaerobic exercise; anaerobic exercise can hone people's endurance and physical quality, can bring people many different benefits, and can also help calf muscles become more full and powerful [19].

Because the foot is the only part of the body that the runner contacts the ground and directly provides power during running, the landing of the foot plays a special role in running technology, especially in the process of contacting the ground. According to the foot strike pattern, the runner's running mode is mainly divided into three types: the hindfoot landing mode, the midfoot landing mode, and the forefoot landing mode. The hind foot landing mode is the initial heel contact with the ground. The study found that more than 85% of middle- and long-distance runners use the rear foot landing mode. The rest of the runners used the midfoot landing mode and the forefoot landing mode. The midfoot landing mode is when the heel and ball of the foot initially contact the ground at the same time, and the forefoot landing mode is when the metatarsal ball initially contacts the ground. Many factors may affect the landing mode, including the type of running shoes that the runner wears, running speed, and running surface. For example, when running on steep slopes, runners tend to use the forefoot landing mode, and when running downhill, they tend to use the hindfoot landing mode. The landing mode of running will affect the transmission of impact force and the change of the lower limb movement biomechanics during running, resulting in different movement patterns of the lower limbs and the conduction of the power chain of the runner, which may cause different locations and rates of sports injuries. Therefore, the landing mode of running is one of the important factors that researchers must consider in the research of running biomechanics, and it is also one of the focuses of current running-related research.

When initially touching the ground, the ankle joints of runners using the forefoot landing mode were slightly flexed, and the ankle joints of the runners using the hindfoot landing mode were slightly dorsiflexion. After initial contact with the ground, the ankle joint of runners using the hindfoot landing mode has a rapid plantar flexion. In contrast, runners who used the forefoot landing mode experienced dorsiflexion in the ankle joint after initial contact with the ground. In addition, runners who use the forefoot landing mode will have greater knee and hip flexion angles. The kinematic change of the ankle joint in different landing modes is one of the important reasons leading to the kinematic change of the knee and hip joints. Compared with runners who use the forefoot landing mode, runners who use the forefoot landing mode have a smaller range of ankle dorsiflexion during the support phase and a larger range of knee and hip joints on the sagittal plane. In terms of the motion of the lumbar vertebrae, compared with runners using the forefoot landing mode, runners using the hindfoot landing mode have a larger range of lumbar spine motion.

At the same running speed, runners who landed on the forefoot showed shorter stride length, higher stride frequency, and shorter ground contact time. This may be because the knee joint flexes more when the runner touches the ground at this time, which shortens the runner's step length. Moreover, runners have more flexed ankles when they touch the ground, which may correspond to increased stride frequency. The increased cadence means that each step has a shorter time to touch the ground.

Muscle activity is caused by nerve impulses. Surface electromyography (EMG), as an effective way to observe muscle activity, can be used to evaluate muscle recruitment, activation, and coordination among muscles. This information about muscle activity obtained by the EMG test can be used to determine the specific internal mechanisms of human biomechanical adjustment. However, the current research on the neuromuscular regulation of the human body when running in different landing modes is relatively limited, mainly focusing on the muscles on the front and back of the calf.

In the time when the ankle plantar flexor muscle (gastrocnemius) is activated before the initial contact with the ground, runners using the forefoot landing mode activate 11% earlier than runners using the hindfoot landing mode. Runners in back foot landing mode are 10% longer. This may have a causal relationship with the structure of the human body. The preactivation of the ankle plantar flexor muscles before contacting the ground can increase the Achilles tendon tension, which in turn helps absorb the impact when contacting the ground. This can not only prepare for contact with the ground but also increase the ability of the tissue structure around the ankle joint to store elastic energy at the beginning of the support phase. Before the foot initially touches the ground, the gastrocnemius muscles are activated, causing muscle contractions. Therefore, for runners using the forefoot landing mode, the impact force upon landing will be immediately counteracted by the gastrocnemius muscle activated earlier and longer, which will help stabilize the ankle joint and stabilize the Achilles tendon load ratio. A medical imaging picture of the plantar flexor muscle is shown in Figure 1.

Compared with runners who used the hindfoot landing mode, runners who used the forefoot landing mode had lower tibialis anterior muscle activity and higher muscle activity on the medial head of the gastrocnemius muscle. For the hindfoot landing mode, there is more muscle activity in the tibialis anterior muscle, while for the forefoot landing mode, there is more muscle activity in the gastrocnemius and soleus muscle.

Many human movements are characterized by the continuous repetition of some basic form of movement (such as walking, running, single-foot jumping, cycling, swimming, and rowing). For periodic exercise, the average speed of the exercise is equal to the product of the average moving distance (such as the step size during running) and the average frequency or rhythm (such as the step frequency during running) of each exercise cycle. In normal human movement, these factors such as speed, distance, and frequency are usually arbitrarily determined or selected by the athlete, rarely fixed or determined in advance, and humans have an amazing ability to change speed, distance, and frequency to adapt to the environment demand. We call the frequency arbitrarily determined or selected by the athlete as the self-selected frequency or suitable frequency.

## 3. Experiments

### 3.1. Data Collection

This experiment selected 20 male students from a sports university. In order to reflect the difference between different running frequencies, the 20 subjects were randomly divided into two groups of low-frequency step and high-frequency step, with 10 boys in each group. The low-frequency step and high-frequency step are divided into three different speeds: low speed, medium speed and high speed.

### 3.2. Criteria for Recruiting Subjects

The criteria for recruiting subjects are as follows: (1) aged between 18 and 30; (2) male; (3) having a running exercise habit, running at least 10 km per week; (4) not receiving special system training. All subjects completed the informed consent form before the experiment to ensure that the subjects were healthy without motor system, neurological diseases, and other major medical histories. In the current state, there was no sports injury and the exercise ability was good. No strenuous exercise was performed within 24 hours before the test, and there was no muscle fatigue.

### 3.3. Experimental Instruments

The experimental instruments used in this study are as follows: infrared high-speed motion capture test system, three-dimensional force plate system, surface electromyography test system, laser speed measurement system, portable ultrasound system, height gauge, weight scale, morphometric ruler, and sports shoes need to be prepared, socks, tights, swimming cap, alcohol cotton ball, double-sided tape, elastic bandage, scissors, and other experimental consumables.

### 3.4. Experimental Methods

The application of a three-dimensional force plate system is studied to collect the ground reaction forces and related indicators in three directions during running, the acquisition frequency is 1000 Hz, and the surface electromyography test system is used to collect the subject's lower limb electromyographic parameters during running, and the acquisition frequency is 2000 Hz. The infrared high-speed motion capture system was used to collect the three-dimensional kinematic parameters of the reflective markers during running, and the instrument acquisition frequency was set to 200 Hz. The acquisition frequency of the experimental instrument is set to achieve frame synchronization between kinematics, dynamics, and surface EMG data. Before the experiment, inform and explain the subject's experimental content and experimental process in detail so that they fully understand and actively cooperate with the test.

The subject naturally stood on the force platform, with both arms raised sideways, feet separated, toes forward, and the positions of each point in the quiet state were marked. The subject then started at a position 13 m straight from the force plate and ran across the 26 m runway at speeds of 2.5 ± 0.2 m/s, 3.25 ± 0.2 m/s, and 4 ± 0.2 m/s, using portable speed measurement. The system monitors the running speed. The subject was not informed of the specific position of the force plate before the test. The subject was required to adjust without steps and step on the force plate with his left foot completely, no reflective landmarks fell off during the acquisition process, and no abnormal EMG signals were used as valid data. Data were recorded corresponding to each test file during the test. Each subject collected valid data 6 times at each speed, and the average value was obtained by excluding the maximum and minimum values.

The data were expressed as mean standard deviation and processed by statistical software. Paired tests were performed on the data of muscle stiffness, tendon stiffness, stiffness of muscle tendon complex, and vertical stiffness of lower limbs in each group. The significance level was *P* < 0.05.

## 4. Discussion

### 4.1. Analysis of Kinematic and Dynamic Parameters at Different Frequencies

#### 4.1.1. Analysis of Kinematic Parameters at Different Frequencies

In this study, the stage where the vertical ground reaction force is greater than 10 N is regarded as the subject stepping on the force plate. According to the dynamic data, find the number of frames at the beginning and end of the left foot support phase, the magnitude of the vertical ground reaction force (the first peak, the second peak), and the number of frames at the time of occurrence; the critical frames of the buffer phase and the kick phase are calculated the support period and relative support period. The vertical ground reaction force value needs to be divided by the subject's weight for normalization to reduce the effect of weight on the force value. Kinematic indicators at different running frequencies are shown in Table 1 and Figure 2.

From Table 1 and Figure 2, it can be seen that when the subjects are running at three speeds, there is no significant difference in step length between the low-cadence group and the high-cadence group, but both show an increase in running frequency and a decrease in step length. The small change trend is observed as follows: at three speeds, the gait period of the high-cadence group is significantly smaller than that of the low-cadence group (*p* < 0.01); at three speeds, the support period of the high-cadence group is shorter than that of the low-frequency group. And it is extremely significant at slow speeds (*p* < 0.01); when the subjects are jogging, the high stride group and the low stride group show a significant difference in the relative support period (*p* < 0.05), and the high stride frequency in the relative support period of the group was significantly shortened, but during the middle and fast running, the low-cadence group and the high-cadence group showed an increase in running frequency and a relative support period. In terms of the relative support period, at the three speeds, the values of slow steps are 40 and 30. It is suggested that the running frequency has an effect on step length, support period, and gait cycle.

#### 4.1.2. Analysis of Dynamic Parameters at Different Frequencies

This study mainly analyzes the effect of different running frequencies on vertical ground reaction forces. After the dynamic data are collected and processed, the number of frames at the characteristic moments of the dynamic data (landing, off the ground, and the time when the maximum ground reaction force occurs) is synchronously converted into the number of frames at the characteristic moments of the kinematics data. Characteristic moments (landing, off the ground, and the moment when the maximum ground reaction force occurs), the lower limb joint angle, the maximum angle of the lower limb joint at the support stage, the minimum angle, and the range of motion (the difference between the maximum angle and the minimum angle) are also analyzed. The analysis of kinetic parameters at different frequencies is shown in Figure 3.

As shown in Figure 3, the first peak of the high-cadence group is larger than that of the low-cadence group when running at slow and medium speeds, and the opposite is true for fast running. The second peak of the high-cadence group is larger than that of the low-cadence group during slow and fast running, but the opposite is true at medium speed, but there is no significant difference.

### 4.2. Analysis of Lower Limb Stiffness and Muscle Vibration Frequency at Different Frequencies

#### 4.2.1. Analysis of Lower Limb Stiffness at Different Frequencies

During running, the person's center of gravity is not always directly above the foot, so when calculating the stiffness, factors such as the speed of the runner, support time, leg length, and angle of the supporting leg and the ground must be considered. This study uses the following formula to calculate the stiffness of the lower limbs during the support phase, the buffer phase, and the active pedal extension phase:

(1) $$\begin{array}{c} k_{\text{leg}}=\frac{F_{\max}}{L-\sqrt{L^{2}-{\left(Vt_{c}/2\right)}^{2}+\Delta y}}. \end{array}$$

Among them, *F*_max_ represents the maximum vertical ground reaction force, *L* represents the leg length, *V* represents the speed, *t*_*c*_ represents the ground time, and Δ*y* represents the vertical displacement of the center of gravity.

The lower limb stiffness analysis at different frequencies is shown in Figure 4.

It can be seen from Figure 4 that during the whole support period, the subjects' stiffness in the lower limbs of the high-cadence group was greater than that of the low-cadence group when running at slow and medium speeds, and the opposite was true during fast running, but there was no significant difference. In the buffer phase, the subjects' lower limb stiffness was lower in the high-cadence group than in the low-cadence group when running at slow and medium speeds, and the opposite during fast running. In the active kick-extension phase, the stiffness of the lower limbs of the high-cadence group was lower than that of the low-cadence group at three speeds.

#### 4.2.2. Analysis of Muscle Vibration Frequency at Different Frequencies

A surface EMG signal is a combined wave composed of many sine waves with different frequencies and amplitudes in a certain time sequence. It is an electrical signal that is continuous in time and amplitude. The analysis of EMG signals includes time domain analysis and frequency domain analysis. This study mainly adopts time domain analysis methods, iEMG, and RMS. iEMG refers to the total discharge of motor units participating in activities in muscles within a certain period of time. The size of the iEMG value reflects the number of sports units participating in the work, the discharge size of each exercise unit, and, to a certain extent, muscle strength. RMS responds to the average level of muscle discharge over time. First, the original data are processed by zeroing, filtering (10–400 Hz), inversion, and low-pass filtering (0–20 Hz), and then iEMG and RMS are calculated. The lower limb stiffness analysis at different frequencies is shown in Figure 5.

From Figure 5, the activity of the rectus femoris, tibialis anterior muscle, medial head of gastrocnemius, lateral head of gastrocnemius, and biceps femoris, rectus, medial head of gastrocnemius, and lateral head of gastrocnemius at slow and fast can be seen; the higher the running frequency, the smaller the RMS trend. Moreover, the RMS of the medial head of the gastrocnemius muscle was significantly different between the low-cadence group and the high-cadence group at medium speed (*p* < 0.05).

## 5. Conclusions

The purpose of this article is to investigate the use of low-intensity lasers in the treatment of muscle strains, analyzing running, muscle conditioning, and lower extremity stiffness.

1. This article analyzes the effects of different running frequencies on various spatiotemporal parameters. The results show that at three speeds, the higher the running frequency, the smaller the step size and gait cycle and the support period. The support period and relative support period of the high-cadence group at the slow speed are significantly lower than those of the low-cadence group. As the speed increases, the support period of the high-cadence group is still smaller than that of the low-cadence group, but there is no significant difference.
2. This article finds that there is no difference in the impact force on the lower limbs at different running frequencies, and the kinematic indexes, such as the displacement of the center of gravity in the vertical direction, have a tendency to change, so it is theoretically inferred that the stiffness of the lower limbs at different running frequencies should be changed. The results calculated in this study are that during the buffer phase, the subjects' lower limb stiffness was lower in the high-cadence group than in the low-cadence group when running at slow and medium speeds, and the opposite was true during fast running. In the active kick-extension phase, the stiffness of the lower limbs of the high-cadence group was lower than that of the low-cadence group at three speeds.
3. This article analyzes the effect of running frequency on muscle tuning and stiffness of lower limbs. It is recommended that people should try to choose a relatively high-cadence at the same speed when running, and runners who are used to lower cadence should appropriately choose professional sports equipment to reduce the risk of sports injuries.

## Figures and Tables

**Figure 1:** Plantar flexor muscle picture.

**Figure 2:** Kinematic indicators at different running frequencies.

**Figure 3:** Analysis of kinetic parameters at different frequencies.

**Figure 4:** Analysis of lower limb stiffness at different frequencies. (a) Support phase; (b) cushioning and stretching.

**Figure 5:** Analysis of lower limb stiffness at different frequencies. (a) Slow and (b) median speed and high speed.

**Table 1:** Kinematic indicators at different running frequencies.

		Low-frequency step	High-frequency step
Slow	Stride (m)	1.9	1.8
	Gait cycle (s)	0.7	0.7
	Support period (s)	0.3	0.2
	Relative support period (%)	40	37

Medium speed	Stride (m)	2.4	2.2
	Gait cycle (s)	0.7	0.7
	Support period (s)	0.2	0.2
	Relative support period (%)	33	34

High speed	Stride (m)	2.9	2.7
	Gait cycle (s)	0.7	0.6
	Support period (s)	0.3	0.2
	Relative support period (%)	30	31

## Data Availability

The data that support the findings of this study are available from the corresponding author upon reasonable request.

## References

[1] Park J. S., Lee H., Choi B. W. (2018). An MG53-IRS1-interaction disruptor ameliorates insulin resistance. *Experimental & Molecular Medicine*.

[2] Bailey J., Mata T., Mercer J. A. (2017). Is the relationship between stride length, frequency, and velocity influenced by running on a treadmill or overground?. *International Journal of Exercise Science*.

[3] Faber I. R., Bustin P. M. J., Oosterveld F. G. J., Elferink-Gemser M. T., Nijhuis-Van der Sanden M. W. (2016). Assessing personal talent determinants in young racquet sport players: a systematic review. *Journal of Sports Sciences*.

[4] Zhu H., Wei H., Li B., Yuan X., Kehtarnavaz N. (2020). Real-time moving object detection in high-resolution video sensing. *Sensors*.

[5] Alsmirat M. A., Jararweh Y., Al-Ayyoub M., Shehab M. A., Gupta B. B. (2016). Accelerating compute intensive medical imaging segmentation algorithms using hybrid cpu-gpu implementations. *Multimedia Tools and Applications*.

[6] Greenup A. J., Bressler B., Rosenfeld G. (2016). Medical mmaging in small bowel crohn’s disease-computer tomography rnterography, magnetic resonance enterography, and ultrasound: “which one is the best for what?”. *Inflammatory Bowel Diseases*.

[7] Rowlands J. A. (2017). Medical imaging: material change for X-ray detectors. *Nature*.

[8] Song H., Brandt-Pearce M. (2013). Range of influence and impact of physical impairments in long-haul DWDM systems. *Journal of Lightwave Technology*.

[9] Krol A., Gimi B. (2016). Medical imaging 2017: biomedical applications in molecular, structural, and functional imaging. *Evaluation and Program Planning*.

[10] Manahov V. (2016). Front-running scalping strategies and market manipulation: why does high-frequency trading need stricter regulation?. *Financial Review*.

[11] Tavera C. A., Ortiz J. H., Khalaf O. I., Saavedra D. F., Theyazn H. H., Aldhyani (2021). Wearable wireless body area networks for medical applications. *Computational and Mathematical Methods in Medicine*.

[12] Wang Q., Lu P. (2019). Research on application of artificial intelligence in computer network technology. *International Journal of Pattern Recognition and Artificial Intelligence*.

[13] Dong Y., Zhang F. (2018). Single car travel time estimation based on running state of low frequency floating car at intersections. *Journal of Geomatics*.

[14] Yamato Y., Hasegawa N., Sato K., Hamaoka T., Ogoh S., Iemitsu M. (2016). Acute effect of static stretching exercise on arterial stiffness in healthy young adults. *American Journal of Physical Medicine & Rehabilitation*.

[15] Howard D., Kenney L. (2017). Energy efficient lower limb prostheses—epsrc. *Impact*.

[16] Xiao F., Ding W. (2019). Divergence measure of pythagorean fuzzy sets and its application in medical diagnosis. *Applied Soft Computing*.

[17] Xie S., Yu Z., Lv Z. (2021). Multi-disease prediction based on deep learning: a survey. *Computer Modeling in Engineering and Sciences*.

[18] Belando Pedreño N., Ferriz-Morel R., Rivas S. (2016). Sport commitment in adolescent soccer players. *Motricidade*.

[19] Tang Y., Fang S., Chen J., Ma L., Li L., Wu X. (2020). Axial compression behavior of recycled-aggregate-concrete-filled gfrp–steel composite tube columns. *Engineering Structures*.

